# A review of MPTP-induced parkinsonism in adult zebrafish to explore pharmacological interventions for human Parkinson’s disease

**DOI:** 10.3389/fnins.2024.1451845

**Published:** 2024-08-07

**Authors:** Emmeline Bagwell, Jessica Larsen

**Affiliations:** ^1^Department of Bioengineering, Clemson University, Clemson, SC, United States; ^2^Department of Chemical and Biomolecular Engineering, Clemson University, Clemson, SC, United States

**Keywords:** zebrafish, parkinsonism, animal models, neurodegeneration, MPTP

## Abstract

Novel work in adult zebrafish, *Danio rerio,* to recapitulate human neurodegenerative disease has proven useful in both pharmaceutical development and research on genetic disease. Due to high genetic homology to humans, affordable husbandry, relatively quick life cycle breeding times, and robust embryo production, zebrafish offer a promising model to test pharmaceutical performance in a high throughput, *in vivo* setting. Currently, most research in zebrafish models of Parkinson’s disease induces the disease in larval or embryonic stage organisms due to ease of administration, with advancement through developmental stages taking only a matter of days. The use of early-stage organisms limits the usability of zebrafish as models for adult disease and specifically age-related neurodegenerative conditions. Recently, researchers have sought to extend the usability of zebrafish into models for Parkinson’s disease. Specifically, 1-Methyl-4-phenyl-1,2,3,6-tetrahydropyridine (MPTP) has emerged as a prodrug that upon injection well-encompasses the biochemical mechanisms and symptomology associated with Parkinson’s disease. By utilizing MPTP in an adult zebrafish model, advancements in Parkinson’s disease research may be achieved. This paper highlights the recent research on this model, comparing it to the human form of Parkinson’s disease.

## Introduction

Parkinson’s Disease (PD) is a neurodegenerative disorder that affects nearly 10 million patients worldwide. Several symptoms of the disorder include neurological-based dysfunction, such as tremor, muscle stiffness, impaired balance, confusion, insomnia, difficulty speaking, and smooth muscle spasms (Armstrong and Okun, 2020; Parkinson’s Foundation, 2024). Several mechanisms are involved in the disease, stemming from both environmental and genetic components. Specifically looking at the pathophysiology of the disease, PD damages the dopaminergic (DA) neurons located in the substantia nigra and the diencephalon, the portion of the midbrain responsible for sensory and autonomic control and processing (Tabrez et al., 2012). Alpha-synuclein, a protein responsible for neurotransmitter and synaptic vesicle trafficking, is overproduced due to the upregulation of the SCNA (synuclein alpha) gene in PD patients. This upregulation causes the accumulation of alpha-synuclein, creating plaques that are responsible for several synucleinopathic neurodegenerative diseases, including PD (Stefanis, 2012). The aggregation of alpha-synuclein plaques at the synaptic cleft eventually prevents neurotransmitter signaling, causing dopamine production to lower. As these plaques continue to accumulate, dopamine transmission occurs at lower levels until the neurons are eventually tagged for apoptosis, or programmed cell death. These plaques can accumulate so rapidly that lysosome cannot control the overload of alpha-synuclein, leading to necrosis (Stefanis, 2012). The pathophysiology and etiology of PD has been extensively reviewed elsewhere (Poewe et al., 2017; Bloem et al., 2021; Zaman et al., 2021).

Due to the several genes and pathophysiological mechanisms at play, PD has no known cure. Current research interests in PD have shifted toward understanding disease mechanisms and identifying pharmaceuticals that could alleviate the excruciating symptoms instead of aiming to treat the cause (Lee et al., 2017). The current gold-standard pharmaceutical treatments for PD are Levodopa (L-dopa) compounds. These compounds mimic the natural pathway intermediate involved in the production of dopamine. Levodopa is often prescribed to patients in intermediate to late-stage PD (Abbott, 2010).

Beyond making treatment difficult, isolation of a common etiology for PD and its complex pathophysiology has made it difficult to model. Research has focused on the use of zebrafish as models for PD research in recent years since the first published zebrafish paper in 2003 (Figure 1). Its exponential growth in use as a PD model is likely due to affordability, accessibility, and replicability (Lam et al., 2005) of zebrafish. In this review article we discuss the relevance of zebrafish as a model organism for human PD, including the reasoning behind its use and its homology to human disease. We specifically highlight the use of neurotoxin MPTP for PD model induction, with a focus on comparing the very few (< 20) studies using this adult-aged model and a call for more uniform protocols. Finally, we end with a discussion on the relevance of testing of explored neurotherapeutics for PD in MPTP zebrafish.

**Figure 1:** Results from a web of science search using the terms “Zebrafish” + “Parkinson’s Disease.” Highlighted here is the exponential growth in the use of Zebrafish as models for Parkinson’s disease from its first published paper in 2003. Note that although there has been a significant amount of growth over the last twenty years, the cumulative number of papers focused on this model is still quite small. MPTP has been used to induce PD since 2005 and has grown in popularity. However, despite the age-related behavior of PD, a very limited number of papers have focused on using MPTP to create PD in adult zebrafish, as highlighted by the gray contribution to the bars each year. When this search was performed, there were only 20 total papers that focused on MPTP in adult zebrafish.

## Zebrafish as a model organism

*Danio rerio,* the zebrafish, is a species that has become popular in research of neurological diseases due to high genetic homology to humans (Mrinalini et al., 2023). Zebrafish belong to the class Actinopterygii, which accounts for over half of all vertebrates (Lawrence and Mason, 2012). Specifically, zebrafish are teleost, meaning that they have complete bone formation in homology with most vertebrates. This homology makes zebrafish excellent in studying neurological diseases, bone diseases, genome editing, and embryonic development. In addition to high genetic homology and conserved biological function, zebrafish reproduce quickly. Development of the embryonic features occurs quickly, within 24 h of fertilization, and the larvae hatch around 2.5 days post fertilization. Specifically, zebrafish can produce 100–600 embryos at a time. This ease of breeding and rapid growth cycle provides researchers with a quick and easily renewable animal model (Chia et al., 2022), unlike traditional mammalian rodent models.

Many researchers utilize the embryonic model of zebrafish in research, as development is modeled well in this early stage (Lee et al., 2017). Specifically, zebrafish can be easily genetically modified during embryonic development. At the embryonic stage, zebrafish can be made fully transparent, leading to an optical advantage, allowing researchers to observe drug effects in real-time as opposed to relying solely on post-sacrificial analysis. However, debate has now turned many researchers of neurodegenerative disease toward sexually mature adult zebrafish (≥ 6 months post fertilization). Due to the nature of neurodegenerative diseases, like PD, occurring primarily in adults over the age of 55, many researchers feel that adult zebrafish maintain developmental homology, including age-related pathology, to humans and should therefore be utilized as a model for these diseases (Chia et al., 2022). Furthermore, it is easy to dose zebrafish with drugs through aquatic environment at all stages, which can provide ease of drug administration and decrease the need for invasive procedures to establish small molecule drug induced disease models (Lam et al., 2005).

Beyond rapid maturation, large clutch sizes, and affordability of husbandry, zebrafish have proven to become a beneficial research animal model of many neurological diseases. The human brain and zebrafish brain may have different configurations, but many homologous and highly conserved structures can be observed in both (Figure 2; Diotel et al., 2020). The same areas implicated by PD in humans are often also implicated in PD models that are created experimentally in zebrafish. These areas include the olfactory bulb, and telencephalon. The olfactory bulb is a dopaminergic-neuron dense region of the brain that is responsible for sense of smell and has a strong relationship with memory and learning (Kozol et al., 2016; Diotel et al., 2020). The telencephalon, or the cerebrum in humans, is one of the largest portions of the brain responsible for all voluntary motor control and most sensory processing. The diencephalon in fish, or equivalent to substantia nigra in humans, is a neuron-dense region of the brain that is responsible for nearly all coordinated movements.

**Figure 2:** Anatomy of the zebrafish brain *vs* a mammalian brain, highlighting proposed homologs. The zebrafish central zone of the dorsal telencephalon (Dc) is proposed to be homologous to the mammalian cortex. The lateral zone of the dorsal telencephalon (Dl) and the posterior zone of the dorsal telencephalon (Dp) are proposed to be homologous to the mammalian Hippocampus (Hipp). While the dorsomedial zone of the dorsal telencephalon (Dm) is proposed to be homologous to the amygdala (Am). Adapted from Source (Lawrence and Mason, 2012). Image copyrighted under CC-BY Version 4.0.

Unlike commonly used invertebrate models, such as *Drosophila melanogaster* and *Caenorhabditis elegans*, *D. rerio* are vertebrate teleosts with orthologs of over 78% of genes found in humans (Ellis and Soanes, 2012). In addition to this high genetic homology, the catecholamine production cascade in this model is highly conserved, making the process nearly identical to humans. In this cascade, dopamine is transported by vesicular monoamine transporter 2 (VMAT2) to signal to other neurons. The dopamine transporter (DAT) at the synaptic cleft on the terminal end of signaling neurons then releases dopamine into the synapse. On the dendritic end of a receiving neuron, the dopamine receptor (D1 Receptor) takes up dopamine, leading to the activation of cyclic adenosine monophosphate (cAMP). cAMP serves as a secondary messenger that allows for signal transduction across neurons in the central nervous system (Lebowitz and Khoshbouei, 2020). Specifically in zebrafish, the neurotransmitter pathways for noradrenergic, serotonergic, histaminergic, and dopaminergic systems are highly conserved and relevant in the discussion of PD (Anichtchik et al., 2003; Tay et al., 2011). Due to the importance of dopamine when studying PD, the production of this neurotransmitter cannot go overlooked. Dopamine is produced from the key amino acid tyrosine. L-tyrosine is hydroxylated by the rate-limiting enzyme tyrosine hydroxylase (TH) to form the precursor to dopamine, L-DOPA (Albarran et al., 2014). L-DOPA can then be converted into dopamine by aromatic amino acid decarboxylase in microglia and in TH-positive neurons (Figure 3).

**Figure 3:** Dopamine production from the amino acid, tyrosine (Albarran et al., 2014). Originally published in A Synopsis of Parkinson’s Disease, 2014 under Creative Commons Attribution 3.0 Unported (CC By 3.0) license. Available from: https://doi.org/10.5772/57102.

Zebrafish models are ideal for high-throughput small molecule screens. This approach can identify new drug candidates and potential therapeutic targets through systematic testing of various compounds for their impact on disease-related phenotypes (Lam and Peterson, 2019). Due to the homology of the catecholamine production cascade, zebrafish models have been developed and used to study compounds and interventions that protect dopaminergic neurons from degeneration. Zebrafish models allow for the study of compounds that modulate dopamine levels and neurotransmitter function (Wang et al., 2021). Potential therapies to explore include drugs that enhance dopamine release, dopamine receptor agonists, or alternative neurotransmitter-based treatments like discovery of medications currently on-market (Martel and Gatti McArthur, 2020). One of the biggest benefits of the zebrafish model is that they are amenable to genetic manipulations. Researchers have explored gene therapy approaches, which have been extensively reviewed elsewhere (Chen et al., 2023; Dumbhare and Gaurkar, 2023; Muleiro Alvarez et al., 2024), to deliver neuroprotective genes to dopaminergic neurons, potentially slowing down their degeneration.

Beyond dopamine production, targeting molecules that improve mitochondrial function and energy production in dopaminergic neurons is a potential therapeutic strategy for PD (Prasuhn et al., 2021) for which zebrafish models have provided invaluable insight (Razali et al., 2021). The process of mitochondrial fusion in dopaminergic and TH-positive neurons is disrupted by PD, leading to higher ROS levels. This eventually results in disrupted cell energy pathways and can therefore cause apoptosis.

Furthermore, targeting the immune response in the brain may help mitigate neurodegeneration in PD (Cai et al., 2022). Neuroinflammation is an important aspect of PD pathology, and zebrafish as a model may aid in identifying anti-inflammatory agents that modulate the immune response within the central nervous system and reduce neuronal damage (Araújo et al., 2022). Neuroinflammation associated with PD includes activated glial cells and increased levels of tumor necrosis factors (TNFs), IFNγ, IL-1, IL-6, IL-2, CXC-chemokine ligand 8 (CXCL8), and monocyte chemoattractant protein-2 (CCL2). Zebrafish have several homologs that are similar to these human cytokines, though very few are identical in function or form. Minimal research looks at these pro-inflammatory cytokines in zebrafish, nor their activation by the prodrug MPTP.

A mechanism that still remains unclear is the mechanism of autophagy involved in the clearance of misfolded proteins, including alpha-synuclein (Fellner et al., 2021). Targeting pathways that enhance autophagy may alleviate the accumulation of toxic protein aggregates in zebrafish and, potentially, in humans. Alpha-synuclein aggregation is a hallmark of PD. However, this pathophysiological aspect of PD is difficult to recapitulate in zebrafish due to the genetic differences in alpha-synuclein (SCNA) in humans, while fish only produce homologs that behave differently (SNCB and SNCG1) (Toni and Cioni, 2015). Alpha-synuclein and beta-synuclein are two related proteins found in the human brain, each with distinct roles and behaviors. Alpha-synuclein is well-known for its involvement in PD, as it forms aggregate structures within neurons in humans, which is a hallmark of the disease (Stefanis, 2012). Zebrafish do not naturally develop alpha-synuclein aggregates, as they lack the SNCA gene (Lopez et al., 2022). However, both humans and zebrafish have the protein-coding gene for beta-synuclein (SNCB). Beta-synuclein is a closely related protein to alpha-synuclein but has different properties (Toni and Cioni, 2015). Unlike alpha-synuclein, beta-synuclein is not commonly associated with PD pathology or Lewy body formation, but it appears to have a protective role against alpha-synuclein aggregation and toxicity (Calabresi et al., 2023). Zebrafish lack alpha-synuclein but have been shown to express the analog proteins beta-synuclein and gamma synuclein (Doyle and Croll, 2022). In knockdown models of zebrafish, beta-synuclein has proven to be directly affiliated with PD-like motor and behavioral issues, making it a relevant marker in modeling of PD (Ninkina et al., 2021). Researchers have studied beta-synuclein in zebrafish models to investigate its functions and its potential protective effects against alpha-synuclein-induced toxicity (Lopez et al., 2022). This research may contribute to a better understanding of the interplay between these two synuclein proteins in the context of neurodegenerative diseases.

Zebrafish models can recapitulate some aspects of parkinsonism due to the anatomical, biochemical, and cellular pathologic similarities to human systems involved, but likely do not fully capture the diversity seen in human PD etiology (Gialluisi et al., 2021). In addition to physiological differences, the mechanism of disease induction in these fish fails to account for the gradual and progressive nature of human PD. Human PD is characterized by progressive loss of dopaminergic neurons and the accumulation of alpha-synuclein over many years (DeMaagd and Philip, 2015). In contrast, zebrafish models often develop symptoms more rapidly after toxin exposure, making it challenging to study the long-term, age-related aspects of PD (Cassar et al., 2020). The pharmacokinetics of drug metabolism, blood–brain barrier characteristics, and drug responses can differ between zebrafish and humans. Therefore, drug testing results may not be directly translatable and must be confirmed in mammalian models before proceeding with development (Cassar et al., 2020; Knap et al., 2023). Despite these differences, zebrafish models offer significant advantages, including rapid development, optical transparency, and genetic manipulability. They are particularly useful for investigating fundamental mechanisms of neurodegeneration and for drug screening (Kim and Jin, 2012). Combining insights from zebrafish with other animal models and human studies will be crucial for a comprehensive understanding of PD. However, due to the homology of catecholamine cascade, there are benefits to the use of neurotoxin models in zebrafish to develop appropriate therapeutics for PD. Specifically, we focus our discussion on the use of a neurotoxin 1-Methyl-4-phenyl-1,2,3,6-tetrahydropyridine (MPTP) as a highly promising model of PD with relatively facile administration in zebrafish.

## MPTP for modeling PD

It can be difficult to recapitulate the full complexity of any human disease in an animal model, but research has identified the use of different types of small molecule drugs that can mimic Parkinsonian symptoms in zebrafish. These different types of drugs to induce Parkinson’s in zebrafish have been explained elsewhere (Makhija and Jagtap, 2014). In this review, we focus on MPTP as a highly promising model of PD with relatively facile administration in zebrafish. The specific MPTP induction of PD has been used since 2004 and has grown in popularity, though its limitations are still up for debate. When a general search was performed from 2001 to 2023, there were only 20 total papers that focused on MPTP in adult zebrafish (Figure 1).

MPTP is a highly lipophilic prodrug analgesic discovered when a batch of desmethylprodine was produced incorrectly (Sallinen et al., 2009). MPTP is metabolized into 1-methyl-4-phenylpyridinium (MPP+) once taken up by astrocytes containing monoamine oxidase-B (MAO-B). The MPP+ metabolite is then taken up by the dopamine transporter (DAT) located on DA neurons. Once this toxin enters the DA neuron, it inhibits oxidative-level phosphorylation in the mitochondria, causing necrosis (Tabrez et al., 2012). This oxidative stress induced by MPTP, which causes neurotoxicity, is similar to a well-known induction of PD in humans (Dias et al., 2013). Mitochondrial dysfunction is a hallmark of PD as well. The process of mitochondrial fusion in dopaminergic and TH-positive neurons is disrupted by Parkinson’s disease, leading to higher ROS levels. This eventually results in disrupted cell energy pathways and can therefore cause apoptosis. The use of zebrafish to study mitochondrial dysfunction also emerging, though MPTP has not been associated with significant changes in mitochondrial function. This mechanism mimics PD by causing necrosis of DA neurons specifically located in the substantia nigra and diencephalon. Dopaminergic neurons are particularly vulnerable to these effects due to their high energy demands and the oxidative environment they operate in Dias et al. (2013). The necrosis of these cells causes the tremor and muscle rigidity characteristic of PD, as well as lowering free dopamine levels and DA neuron numbers in these regions (Anichtchik et al., 2003). The loss of dopaminergic neurons in the substantia nigra and other regions of the brain result in motor symptoms that resemble those seen in PD, such as bradykinesia, tremors, rigidity, and postural instability. The toxic mechanism of MPTP and its conversion to MPP+ serves as a valuable tool for creating animal models of PD in research, as it recapitulates some of the key pathological features of the condition (Mat Taib and Mustapha, 2020). However, it is important to note that the progression of MPTP-induced parkinsonism is often more rapid and severe than that of idiopathic Parkinson’s disease in humans, and MPTP is not considered a causative agent of idiopathic Parkinson’s disease in human patients.

Despite its downfalls, MPTP has emerged as a highly beneficial drug product in research of PD due to its pharmacodynamic behavior in neural tissues (Vaz et al., 2018). MPTP is beneficial due to its ability to recapitulate both effects on catecholaminergic production as well as behavioral and motor deficits. However, despite this fact most MPTP zebrafish models still involve the use of fish in early stages of development. One of the leading reasons for the use of the zebrafish embryonic model of PD is ease of induction, as MPTP can simply be dissolved to appropriate dilutions in tank water. The embryonic stage zebrafish are able to absorb the neurotoxic MPTP through their gill capillaries, causing permanent neurological deficits within hours. Several researchers have utilized this method and allowed the fish to reach sexual maturity after incubation in MPTP during the larval stage of development (Vaz et al., 2018; Razali et al., 2021). Figure 1 highlights the growing interest in establishing an adult model of disease over the last 20 years; these adult zebrafish may more adequately recapitulate human aging processes and enable a more in depth understanding of human PD.

MPTP, combined with the use of adult zebrafish, have led to animal models that encompass some quantifiable and observable changes associated with human PD (Anichtchik et al., 2003). However, despite the growth of this field, the use of MPTP in adult zebrafish still lacks universally accepted and uniform protocols, as delivery routes and doses for MPTP, tissue analysis methods, and movement analysis methods vary widely (Vaz et al., 2018). Below, we highlight the use of MPTP in adult zebrafish as a model for PD by comparing the presentation of PD in these animals versus what is observed in human patients (Vaz et al., 2018). We aim to identify best practices associated with model development and provide guidance for the field. Although not a perfect recapitulation of disease, this model has the potential to expand upon our knowledge of PD and identify new treatment modalities for human clinical trials.

## Adult MPTP- treated zebrafish as models for PD

Table 1 highlights the current experimental papers focused on the use of MPTP in adult zebrafish to induce models of PD. It becomes quite clear with the lack of experimentation being done on adult zebrafish that there is a lack of consistency in the procedural set up and the fish characteristics, which may be contributing to a lack of consistency in both the behavioral and neurochemical observations. As MPTP with zebrafish becomes an increasingly popular research topic for animal models of PD, several research groups have produced foundational knowledge that could be used in the development of a more uniform model. There is a lack of consistency in the age, genders, and strain of zebrafish being used in experimentation. In the context of zebrafish, “adult” typically means reaching sexual maturity which happens around 3 months (Singleman and Holtzman, 2014). The aging of zebrafish is being explored and is linked to functional changes (Kishi, 2004), which could impact study outcomes and make comparison of findings irresponsible.

**Table 1:** A summary of current literature on adult-induced parkinsonism in zebrafish using MPTP.

Fish line	Procedural set up		Fish characteristics		Behavioral analysis		Neurochemical analysis			References
	Injection route	MPTP concentration	Age	Gender	Locomotor activity	Cognitive function	Dopamine	Tyrosine Hydroxylase (TH)	Synuclein	
Transgenic zebrafish Tg(dat:eGFP); Tg(dat:tom20 MLS:mCherry)	Cerebroventricular microinjection (CVMI)	10, 25, 35, 100 mM	10 months	-	47% decrease in avg. velocity and distance 51% increase in freezing	marked motor and olfactory function decline	65% of dopaminergic neuron mitochondria fragmented	47% loss in occipital lobe 25% loss in periventricular pretectal nucleus 41% low in telencephalon	-	Kalyn and Ekker (2021)
AB zebrafish	Intraperitoneal (IP)	Single dose or double dose of 50 μg	6 months	50:50 M:F	decreased distance by 25% in single dose and 68% in double dose	-	-	TH reduced, but not significantly	Decreased SCNA and increased α-synuclein after 2 doses	Sarath Babu et al. (2016)
Outbred and AB Zebrafish	Intramuscular (AM)	20, 40, 60 or 80 mg/kg	Adult	M:F	20% decrease in distance and 80% decrease in velocity 9 days after injection	Decreased tank exploration	Sustained decrease of 30%	TH decrease shown via western blot	-	Anichtchik et al. (2003)
Wild Type (WT) outbred long-fin strain	IP	0, 50, 100, 200 and 400 μg in 1 %DMSO/PBS	~ 1 year old	50:50 M:F	No locomotor deficits observed	Y-maze showed that spontaneous alternation behavior decreased	Linked social behavior to dopamine D3 receptor agonism in zebrafish	-	-	Bashirzade et al. (2022)
AB Zebrafish	IP	200 μg/g body weight	3 to 4 months	-	Statistically decreased velocity and distance at 24 h post injection	Increase in freezing bouts that remained high for 96 h	-	Fewer expressed TH+ neurons in substantia nigra	-	Razali et al. (2022)
Zebrafish from a local aquarium	IP	100 μg/g	5 months	-	Significant decrease in length and distance traveled 24 h post injection	Significant increase in freezing + significant decrease in rapid movement	Fold change in dopamine expression of 0.5	-	-	Selvaraj et al. (2019)
WT zebrafish	IP	225 mg/kg	< 8 months	-	3x decrease in distance traveled and mean speed	50% decrease in number of line crossings	3-fold decrease in dopamine content from 900 to 300 ng/g	-	-	Nellore et al. (2013)

The method and concentration for dosing MPTP became a point of debate due to the bioavailability and safe dose that could be of therapeutic importance. Clearly, from Table 1, the great majority of MPTP injections performed in adult zebrafish are intraperitoneal (IP) (Sallinen et al., 2009; Tabrez et al., 2012; Dias et al., 2013; Makhija and Jagtap, 2014), with one using a direct-to-brain approach via cerebroventricular (CV) administration (Kalyn and Ekker, 2021) and one exploring an intramuscular (IM) route (Anichtchik et al., 2003). These routes all lead to different pharmacokinetic profiles for MPTP, with bioavailability expected to vary significantly, but in all cases MPTP is able to affect neurologic tissue. It does appear that the direct-to-brain, CV injection led to the greatest decrease in TH, which may mean that this injection route leads to the most MPTP activity in the brain. With regards to dosing, MPTP concentrations also varied, even within IP-injected studies. Omar et al. (2023) determined toxic IP-injected MPTP doses, which had them settle on injections of 100 μg/g, but other groups have still explored up to double this dose (Razali et al., 2021).

Due to the broad spectrum of symptoms associated with human PD, MPTP zebrafish studies have focused on assessing the fish for both their behavioral and neurochemical changes. One of the most consistent findings in the adult zebrafish MPTP model confirms that locomotor changes mimic human PD. Decreases in both average velocity and average distance traveled during study periods were consistently observed regardless of MPTP injection route, MPTP concentration, or precise fish age. When assessments were performed, cognitive function declines were also consistently observed. Specifically, cognitive tests have been performed to identify freezing periods (Selvaraj et al., 2019; Kalyn and Ekker, 2021), similar to human bradykinesia, behavioral alterations, like changing swimming patterns (Anichtchik et al., 2003; Nellore et al., 2013) and decreasing in exploration of new spaces (Bashirzade et al., 2022). Overall, these studies all conclude that adult zebrafish experience similarities in movement related symptoms, specifically bradykinesia-like, regardless of method of administration of MPTP.

Though much of the groundwork establishing locomotor activity change and behavioral change has been replicated by several groups, assessing for neurotransmitter and gene expression is still being discovered. Dopamine expression, either the neurotransmitter form or dopamine transporter expression, have become an increasingly popular hallmark to assess for when discovering the underlying mechanisms of PD. After imaging of neurological tissue, counting the number of dopaminergic (DA) neurons has become a quantifiable way to determine a decrease in MPTP-treated zebrafish (Matsui and Sugie, 2017). Some studies did quantify DA neuron losses, while others quantified changes in dopamine expression, with three papers seeing between 30 and 50% decreases in detectable dopamine after MPTP injection. Similar observations with TH are observed, with reductions in both number of TH+ neurons and in TH levels. However, around half of currently published assessments do not look at any quantification of dopamine or TH, despite their marked importance in human PD. A second major component associated with the pathophysiology of PD is the aggregation of the neural protein alpha-synuclein. These aggregates, though a known mechanism of PD, have minimal *in vivo* research with zebrafish models. Though zebrafish do not have genetic markers capable of producing alpha-synuclein, they are able to produce sister proteins beta-synuclein and gamma1-synuclein. Though research on the function of these other synuclein proteins is still emerging in zebrafish research, many studies have concluded that these functions are similar to alpha-synuclein in human adults, as highlighted above.

Although clearly an emerging model, MPTP-induction of PD in adult zebrafish demonstrates a lot of promise. Because zebrafish experience aging related phenomena, it may be significant to develop a consensus of best practices regarding age at MPTP injection. Because the ultimate cognitive and functional decline, as well as dopaminergic and TH level decline is consistent regardless of MPTP dose or injection method, these factors do not currently appear to be significant when developing a PD model. However, as this model matures it may be significant to delineate biochemical changes associated with specific MPTP doses in order to study the various stages of neurodegenerative progression which could lead credence toward therapeutic discovery and development for PD.

## Conclusion

Though the affordability, mass sample size, and high genetic homology makes the zebrafish model promising, much work still is required to bridge the gaps in knowledge. PD is a widespread neurodegenerative disorder affecting millions of individuals worldwide, manifesting with a range of debilitating symptoms, including tremors, muscle stiffness, impaired balance, cognitive impairment, and more. The disease’s complex pathophysiology involves genetic and environmental factors, ultimately resulting in the degeneration of dopaminergic neurons in critical brain regions. Although zebrafish offer a promising model for PD research due to genetic homology, the study of pro-inflammatory cytokines, reactive oxygen species, and mitochondrial dysfunction, all hallmarks of human PD, remains underexplored in this model.

As MPTP with zebrafish becomes an increasingly popular research topic for animal models of PD, several research groups have produced foundational knowledge pertaining to creating a uniform model. The method for dosing MPTP became a point of debate due to the bioavailability and safe dose that could be of therapeutic importance. Two injection routes, IP and CVMI, provided physiological changes that mirrored some of those seen in human PD patients. Research in this model has focused on assessing cognitive function, locomotor activity, dopamine expression, and TH expression. One of the most well-established findings in the adult zebrafish MPTP model confirms that cognitive function declines after a working dose of MPTP. Behavioral tests assess for freezing periods, velocity, and behavioral alterations and have established that zebrafish dosed with MPTP exhibited behavioral deficits and cognitive decline. There has, thus far, been less consistency in other observed neurochemical PD-related changes, as summarized in Table 1.

The pursuit of PD treatments has shifted toward alleviating symptoms, as a cure remains elusive. However, the emergence of zebrafish as a valuable model organism offers hope for advancing our understanding of PD mechanisms and potentially identifying new treatment modalities. Overall, zebrafish hold great promise as a versatile and cost-effective model organism for studying neurological disorders, including PD. The continued exploration of zebrafish models, coupled with a better understanding of PD pathophysiology, may ultimately lead to new insights and potential therapies for this challenging disease.

## Author contributions

EB: Writing – original draft, Writing – review & editing. JL: Funding acquisition, Supervision, Writing – original draft, Writing – review & editing.
